# A Rare but Significant Cause of an Enlarging Neck Mass: A Case Report of Primary Thyroid Lymphoma

**DOI:** 10.4021/wjon515w

**Published:** 2013-07-15

**Authors:** Scott Goodwin, Kim Carmichael

**Affiliations:** a Division of Endocrinology, Metabolism, and Lipid Research, Washington University in Saint Louis, USA

**Keywords:** Thyroid lymphoma, Large diffuse B-cell lymphoma, Autoimmune thyroid disease

## Abstract

Primary thyroid lymphoma is a rare form of non-Hodgkin’s lymphoma that typically presents as a rapidly enlarging goiter in patients with a history of autoimmune thyroid disease. We present the evaluation, pitfalls in diagnosis, and treatment of a 49-year-old woman with diffuse large B-cell primary thyroid lymphoma presenting with airway obstruction.

## Introduction

A new neck mass is a relatively common problem with a rather broad differential. Evaluation of this finding must be approached in a thorough and disciplined manner in order to effectively rule out rare, but quite serious, pathologies. Primary thyroid lymphomas are rare causes of a goiter that can have a poor prognosis if not discovered and treated efficiently. Unfortunately, the diagnosis of this form of non-Hodgkin’s lymphoma can be difficult due to the non-specific physical exam, laboratory, imaging and histopathological findings. A higher index of suspicion is needed for this diagnosis so that non-routine, but appropriate, analysis is performed.

## Case Report

A 49-year-old woman presented with a rapidly enlarging neck mass with stridor and respiratory distress. Three months prior, she was noted to have a goiter and elevated serum thyrotropin (TSH) by her primary care physician. She was diagnosed with primary hypothyroidism, treated with levothyroxine 75 µg/d, and had a fine needle aspiration of the neck mass which reportedly showed benign thyroid characteristics. She was treated with a course of corticosteroids for presumed thyroiditis.

Despite the corticosteroids, she noted continued growth of her neck mass with accelerating symptoms of odynophagia, dysphagia to solids, hoarse voice and eventual dyspnea, with subsequent transfer to our care. She had been unable to take the prescribed levothyroxine due to difficulty with swallowing. There was no history of radiation to her neck. She had no significant past medical history or family history of thyroid disorders, autoimmune diseases, rheumatic diseases, or cancer, but she had a 30-pack-year history of tobacco use. She denied any recent weight changes, temperature intolerance, fevers, chills, or night sweats.

On exam she was afebrile and hemodynamically stable. Her weight was 41 kg. She spoke in a soft, hoarse voice of 5 - 7 words per sentence. Her eyes were without proptosis or periorbital myxedema. Her eyebrows were fully intact. She had moist mucus membranes without evidence of thrush. Her thyroid was large, approximately 120 grams, nontender to palpation, asymmetric and had irregular texture. There was no palpable anterior cervical, clavicular, or axilliary lymphadenopathy. Her breath sounds were clear to auscultation in her chest, although she did have mild upper airway stridor. Heart was regular. Extremities were free of edema. Her skin was mildly dry, but there were no rashes. Her deep tendon reflexes were slightly delayed.

Laboratory included: TSH 36 µIU/mL (normal: 3.5 - 5.5); free thyroxine 0.6 ng/dL (0.9 - 1.8); thyroid perioxidase (1,524 IU/mL) and thyroglobulin antibodies (> 500 IU/mL) were significantly elevated. Complete blood count revealed a normal leukocyte count with no premature forms, hemoglobin 11.4 g/dL (normal: 12.1 - 15.1), mean corpuscular volume 93 (normal: 80 - 97), and a normal platelet count. Erythrocyte sedimentation rate was 13 mm/hr (normal: 0 - 20). Chemistry panel normal. Lactate dehydrogenase 563 IU/L (normal: 100 - 250).

Computer tomography imaging with intravenous contrast (Fig. 1) was obtained and demonstrated a homogeneously enhancing solid mass, measuring 8 cm × 9 cm × 15 cm, arising from the thyroid gland with circumferential encroachment on the central airway narrowing the tracheal lumen to 6 mm at the level of the clavicles. No satellite lesions or lymphadenopathy was noted. No lytic or blastic bony lesions were seen.

**Figure 1:** CT scan of the neck with intravenous contrast revealing a large mass originating from the thyroid gland with compression of surrounding structures. No obvious lymphadenopathy, satellite lesions, or bony lesions.

Fine needle aspiration and ultrasound-guided large bore core needle biopsy revealed sheets of atypical lymphocytes with very little colloid and infiltrative lymphocytes of varying sizes. A Ki-67 showed a high proliferative index of 60%. Flow cytometry showed 22% CD19+ B-cells lacking expression of light chains, moderate expression of CD20 and negative expression of CD5, CD23, and CD10, all consistent with an aggressive diffuse large B-cell lymphoma (DLBCL) with high proliferation index.

Whole body positron emission tomography revealed metabolic activity in multiple cervical and supraclavicular lymph nodes as well as intense activity within the thyroid gland, classifying her thyroid lymphoma as DLBCL-type, stage IIE of the Ann Arbor staging criteria with an International Prognostic Index score of 2.

Combined chemotherapy and directed radiotherapy resulted in near complete relief of her neck symptoms after the first cycle. She completed 3 cycles of rituximab, cyclophosphamide, hydroxydaunorubicin, oncovin, and prednisone (R-CHOP) followed by 40 Gy locally directed radiotherapy. She did not require thyroidectomy or other surgical resection. Follow-up imaging 24 months after completion of therapy demonstrated complete resolution of her neck mass and no significant lymphadenopathy (Fig. 2). She remains without neck or B-type symptoms. Her anemia has resolved and her LDH is normal. She is clinically and biochemically euthyroid on levothyroxine 75 µg/day.

**Figure 2:** CT scan of the neck/chest with intravenous contrast performed 24 months after treatment demonstrating complete resolution of the thyroid mass and no abnormal lymphadenopathy.

## Discussion

Primary thyroid lymphoma is an exceedingly rare malignant tumor, representing only 1-5% of all thyroid cancers [1-3] and only 2% of extranodal lymphomas [4]. Thyroid lymphomas most commonly occur in middle to older aged individuals with a female predominance. Some authors have reported that these tumors occur almost 3 times more often in women than men [5].

The normal thyroid gland contains no lymphoid tissue. However lymphocyte infiltration into the thyroid can be seen in various pathological conditions, most notably in autoimmune thyroid disease such as Hashimoto’s thyroiditis. Some authors have postulated that thyroid lymphoma may actually arise from the autoimmune thyroiditis transition to mucosa-associated lymphoid tissue (MALT). The transition of MALT to other more aggressive lymphomas with poorer prognosis, such as diffuse B-cell lymphoma, has been observed [3, 6, 7]. In fact, preexisting autoimmune thyroiditis is the only known risk factor for primary thyroid lymphoma. Patients have positive thyroid antibodies (TPO, anti-thyroglobulin, anti-microsomal) in 50-100% of cases of thyroid lymphoma [5, 7, 8]. Not surprisingly, the risk of thyroid lymphoma is 60 times higher in patients with Hashimoto’s thyroiditis than in patients without thyroiditis [7, 8].

The most common initial presenting symptom of thyroid lymphoma is a rapidly enlarging neck mass (goiter) that frequently causes compressive symptoms. Therefore, thyroid lymphoma should be in the differential of any patient who presents with an enlarging neck mass over few to several weeks, especially if they also have a history of Hashimoto’s thyroiditis.

Despite the rarity of this diagnosis, a clinician should maintain a high degree of suspicion for thyroid lymphoma in patients with a rapidly enlarging goiter as the diagnosis remains difficult due to nonspecific physical exam findings, laboratory assessments, and neck imaging. Ultrasound images of thyroid lymphoma commonly show a nonspecific goiter with pseudocystic lesions [9], also commonly seen in patients with Hashimoto’s thyroiditis. Additionally, cytology from fine needle aspirations of the goiter in thyroid lymphoma shows abundance of monomorphic lymphoid cells, a finding also common in Hashimoto’s thyroiditis. In thyroid lymphoma, the lymphocytes are in large number and typically display uniform size and character [5], in contrast to a greater variability seen in Hashimoto’s thyroiditis. These subtle differences can lead the clinician to perform additional testing, such as core needle/open biopsy and flow cytometry analysis.

Treatment of thyroid lymphoma depends greatly on the subtype (for example, MALT, DLBCL) and stage. Non-aggressive, low stage tumors (namely MALT-1E) can be treated with thyroidectomy [10]. However, surgery is of little value in patients with more advanced lymphoma (stage II-IV) and/or patients with a more aggressive lymphoma subtype [3, 5]. The mainstay of therapy rests in chemotherapy with or without adjuvant radiotherapy, as in other types of non-Hodgkin’s lymphoma.
